# Digital Transformation and Firm Performance in the Context of Sustainability: Mediating Effects Based on Behavioral Integration

This article has been retracted.

**DOI:** 10.1155/2022/8220940

**Published:** 2022-09-30

**Authors:** Wei Tang, Shuili Yang

**Affiliations:** ^1^School of Economics and Management, Xi'an University of Technology, Xi'an, 710054 Shaanxi, China; ^2^School of Accounting and Finance, The Open University of Shaanxi, Xi'an, 710119 Shaanxi, China

## Abstract

In order to promote digital industrialization and industrial digitalization, promote the deep integration of digital technology and real economy, and enable the transformation and upgrading of traditional industries and performance improvement, the method of digital transformation and enterprise performance under the sustainable background based on the mediation effect of behavior integration is proposed. This article adopts the case study method, takes Group A as the research object, and excavates the internal and external motivation and transformation path of Group A's digital transformation by combining the theories of organizational change, process reengineering and enterprise life cycle. Combined with the relevant indicators of four dimensions of balanced scorecard, this article deeply studies the impact of digital transformation on the performance of Group A and its internal mechanism. The experimental results show that compared with Group A before digital transformation, the growth rate of gross margin in 2013 was significantly accelerated, and it has always been in a state of stable growth. However, it fell in 2017, when the year-on-year growth rate of the company's total operating revenue and costs was more than 50%, but the actual growth rate of operating expenses was about 5% higher than that of operating revenue. The comprehensive score of Group A's financial performance in 2012 was very low, which did not achieve the desired effect either in terms of growth ability or business strength. In such a situation, Company A began to implement digital transformation, the overall IT system was to carry out a comprehensive reconstruction in the inventory management mode to implement a new model of “sales to production”. By 2013, the financial performance composite score had increased significantly. The comprehensive score of Group A's financial performance in 2012 was very low, which did not achieve the desired effect either in terms of growth ability or business strength. Under such circumstances, Company A began to implement digital transformation, and the overall IT system was comprehensively reconstructed. In the inventory management mode, the new mode of “sales to production” was implemented. By 2013, the financial performance composite score had increased significantly. *Conclusion*. Digital transformation drives the performance improvement of Group A. From the financial perspective, digital transformation has improved the profitability and operation capacity of Group A.

## 1. Introduction

In today's world, the Internet is spreading all over the world and digital technologies are changing faster and faster. The content of people's daily life can be transformed into information and data. In recent years, there is a “happy cloud” that has been written as “artificial intelligence” and is ready to release everything from the emergence of the Industrial Internet to the Internet itself. Scientific and technological tools that get the right information in time and solve problems quickly, smartly, and accurately are constantly updated. Based on information and modern communication network technology, this digital technology continues to enter our lives like bamboo after rain. Technology has not only made people's daily work and life better and more efficient but also started a wave of changing and renewing international business models, developing and optimizing the entire value chain, and radically changing the form of finance [1]. The Digital Economy is a business that follows the development of the times. It is obvious that the global economic development is slow. With the development of science and technology and changes in people's lives, new elements that affect economic growth are constantly emerging. Despite the challenges and changes, the development of the digital economy remains unstoppable in many countries. As the leader of the global digital economy, the digital economy of the United States exceeded 13.1 trillion USD in 2019 and is still the world leader. In recent years, China's economy has grown rapidly, and China has attached great importance to the development of the digital economy. The scale of China's digital economy reached 5.2 trillion US dollars in 2019, ranking second in the world [2]. In addition, South Korea, India, Canada, Italy, and many others have advanced the digital economy, and the growth of the digital economy is covering the world. How to use modern technology effectively, how to change and adapt ourselves to changes in the external environment, how to improve and fix the importance of value creation, and create new ways of value creation—many problems need to be fixed urgently and need a solution [3].

## 2. Literature Review

Fu believes that digital transformation can improve the dynamic capability of enterprises, then improve the innovation performance level, and increase the R&D innovation capability of enterprises. Individual forgetting and entrepreneurship orientation play an intermediary role between digital transformation and dynamic capability of enterprises [4]. Ng and Yee Found that data-driven reform of enterprise product research and development mode can improve enterprise innovation performance and change product innovation research and development mode through data enhancement driven, data system mixed driven, and system innovation driven to achieve innovation in enterprise research and development process [5]. In terms of research on small and medium-sized manufacturing enterprises, Yin et al. studied the relationship between the implementation of digital transformation strategy and the performance of new product development [6]. With the improvement of enterprises' R&D and innovation capacity, the improvement effect of digital transformation on the performance of development is more obvious [7]. Kesavan et al. conducted an empirical study on panel data and found that enterprise innovation performance can be improved by improving the digitalization level of specific regions, and the influence of regional digitalization level on enterprise innovation performance shows an “inverted U-shaped” relationship, which also revealed that one of the ways to improve enterprise innovation performance is to improve the construction level of regional digitalization platform and strengthen the application ability of digital technology [8]. Shahbaz et al. concluded through empirical study that compared with enterprises that did not implement “Internet +”, enterprises that implemented “Internet +” increased their earnings per share by 31% on average and their return on assets by about 24% [9]. With the continuous improvement of digital technology, enterprises have enhanced their capabilities in data acquisition, storage, analysis, and other aspects and created considerable sales performance [10]. Weber et al. analyzed the transformation of Customer Management of SPD Bank and found that the construction of a digital interactive platform in traditional industries fully reflects the Internet thinking, which can concentrate users and continuously interact with each other. One of the ways to improve the core competitiveness of enterprises is to force value innovation, while the transformation and upgrading of customer management in traditional industries requires the innovation mechanism of value creation [11].

## 3. Research Methods

### 3.1. Motivation of Group A's Digital Transformation

As the world economy continues to slump, coupled with the rapid development of Internet technology, many companies are eager to find an effective way to develop in today's situation. In the current domestic environment, whether it is to improve the overall quality of talents, enhance the value of products, reduce operating costs, or expand marketing channels, there is no stable profit model and there may be certain risks, so executives of enterprises dare not take risks [12]. When the digital economy boomed, digital transformation strategy was launched, which is supported by national policies as well as the successful experience of leading enterprises. Therefore, digital transformation has become a good choice for enterprises, as shown in Figure 1.

However, due to the differences in industry, development stages, and awareness level, enterprises in various industries have different reasons for implementing digital transformation. As a traditional household appliance manufacturing enterprise, Group A carries out digital transformation mainly for the following reasons:(1) to meet the needs of the development of the digital economy era, (2) support from national policies, (3) enhance the core competitiveness of enterprises, and (4) reduce product costs and meet the diverse needs of customers.

### 3.2. The Process of Group A's Digital Transformation

The nearly ten-fold growth of Group A's market value is the result of its digital transformation over a decade. So far, Group A's digital transformation has gone through five stages: digitalization 1.0, “Internet +”, digitalization 2.0, industrial Internet, and comprehensive digitalization [13].

### 3.3. The Path of Group A's Digital Transformation

#### 3.3.1. Reconstructing the IT Architecture

In order to realize effective control and management of the whole business process, Company A implemented digital transformation since 2012, completed the manufacturing and control of various kinds of products by using the “632” project, and gradually reconstructed the IT system. It unified all the information in the company and established six sets of different operating systems to apply to each production link of the company in order to smooth the information chain of supply, production, and marketing of the company and complete the interaction between the company and the upstream and downstream of the value chain. All the development end of the company adopts PLM technology to assist the company in completing design and technology development projects [14]. Through ERP, APS, and MES, the company's production process is controlled and optimized. Through SRM system, product supply link is implemented overall control. CRM system is used to provide after-sale service to customers, thus improving the after-sale service effect. Next, the FMS platform is used to coordinate and manage the financial data of the enterprise. And HRMS platform is used to carry out enterprise personnel management. At the same time, BI platform is used to obtain and sort out all aspects of information, thus providing some important basis for enterprise investment and decision-making. Finally, two information management portals, MIP and MDP, are used to complete the sharing of information resources within the enterprise and achieve the purpose of unified operation and management of the enterprise through the collaborative work among various departments.

#### 3.3.2. Change the Original Production and Marketing Mode

The traditional manufacturing mode of home appliance industry is mainly based on channel inventory, that is, production first and then sales. In this way, due to the mismatch between production and sales, enterprises are unable to accurately predict the demand, which is prone to the phenomenon of mismatch between supply and demand, overstocking of unsalable products and shortage of best-selling goods. To this end, Company A began to focus on customers and changed mass production into targeted production according to customer needs through T+3 mode [15]. This mode of production and marketing has successfully improved the quality of product manufacturing and the degree of production automation information, realized the up-down connection of supply chain, and realized the sharing of information resources, enabling Group A to play a synergistic effect in production, manufacturing, distribution, and other links, shorten the product development cycle, reduce inventory pressure, and speed up turnover efficiency.

The T+3 order mode consists of four stages in total, as shown in Figure 2, and each stage is 3 days. T is the time when customers place orders. At this stage, merchants communicate with customers and place orders on the cloud marketing platform according to customers' requirements. T+1 is the cycle of material preparation, during which regional agents and distributors allocate and replenish raw materials through CCS channel coordination system. T+2 is the product processing cycle, in this stage, the provincial city operation center carries out flexible production and warehousing according to the order. T+3 is the cycle of logistics distribution and transportation. The logistics network established by ourselves can realize direct distribution to the manufacturing workshop and shorten the turnaround time of products in the intermediate link. T+3 customer order mode requires good cooperation in all aspects of the whole production process. In the early stage of raw material preparation, the supplier must make a timely response to the terminal demand. Group A has successfully realized the transformation from traditional production to sales.

#### 3.3.3. Expand Sales Channels

In the network era, the traditional marketing methods have been unable to meet the needs of consumers. The retail industry should be driven by customer demand, the online and offline network integration should be accelerated, and the operation system of the retail industry should be reshaped according to the needs of different consumer groups. After T+3 mode, Zhaopin platform deeply promoted the reform of channel logistics, completed the implementation of the strategy of warehouse distribution nationwide, and provided strong support for expanding sales channels. The launch of cloud marketing APP further simplified the sales channel, successfully launched mobile payment, product consulting, and other functions, making the information transmission channel more efficient and transparent. In the agent mode, cloud marketing APP will become the mall mobile network platform between distributors and agents so as to achieve the transparency of the whole channel information. Under the operator management mode, cloud marketing APP directly combines logistics distribution and inventory. Operators do not need to prepare goods by themselves, but only undertake channel business operation. Dealers can directly conduct financing, logistics distribution, and financial exchanges with central enterprises, thus achieving a truly flat channel level [3]. At the same time, customers' purchasing experience is enhanced, which creates an e-commerce purchasing and marketing network platform connecting upstream and downstream for tens of thousands of enterprise distribution end users, which makes the interconnection between the company and the internal sales channel more convenient, and it also helps us to quickly understand the sales and inventory situation of the channel so as to get closer to the market and improve the efficiency of the sales channel. It can realize enterprise digital distribution service management more quickly.

## 4. Result Analysis

Digital transformation refers to the use of information technology to reshape an organization's IT architecture and business architecture. In 2012, Group A reconstructed its entire IT system, abandoning the traditional “large-scale and low-cost” development mode, which can be said to be the most thorough change in the whole development process. Therefore, the chairman of Group A took 2012 as the beginning of its digital transformation. In the following years, he has been actively laying out the road of digital transformation, and has undergone great changes in production, sales, and other aspects. In order to better understand the performance changes of Group A before and after digital transformation, this article adopts the four dimensions of the balanced scorecard to select the relevant data of Group A from 2010 to 2020 for analysis. Since the effect of transformation has a certain delay, the data of Group A in 2013 is used as the watershed before and after the transformation. 2013 to 2020 is the period of digital transformation, and the impact of transformation on performance can be evaluated by analyzing the indicators of Company A [16]. Then, through horizontal comparison with the industry average level, it can be judged whether the change of Company A's performance is an industry trend [17].

When analyzing the financial dimensions of Group A before and after its digital transformation, this article selects relevant financial indicators in profitability, operating capacity, debt paying capacity, and development capacity.

### 4.1. Profitability

It generally refers to the size of the company's profit ability in a certain period of time, which is a relative concept. The higher the profit margin, the stronger the profitability, and vice versa. Company A's operating performance can be reflected from its profitability. This article analyzes the profitability of Group A by ROE and net profit rate on sales.

First, return on equity is calculated according to the following:

(1) $$\begin{array}{c} \text{ROE}=\frac{\text{Net profit}}{{\text{Shareholders}}^{\text{'}}\text{ Equity}} \end{array}$$

This index is mainly used to reflect the benefits generated by the use of the company's own funds in the process of operation. As shown in Figure 3, the line chart drawn based on the data shows that before 2013, the ROE of Company A was declining, but after the transformation, it began to improve from 2013. This is mainly due to the fact that Group A reconstructed the entire IT system in 2012, eliminated the traditional management mode, reduced costs, improved return on assets, and improved profitability [18]. However, in 2016, affected by the growth of market capital scale, the capital scale of Company A has exceeded 30% year-on-year growth rate for two consecutive years since 2016, leading to a decline in the growth rate of ROE. However, the growth rate declined due to the impact of the 2020 pandemic. However, in general, although the index fluctuated during the decade, the main reason for the decline was the influence of M&A factors and the temporary mismatch between revenue and earnings.

A horizontal comparison between the ROE of Group A and the industry average shows that the ROE of the home appliance industry has been growing steadily before 2014. However, the ROE of Company A declined rapidly. After 2014, the return on equity of the home appliance industry is not stable. By actively building new product research and development bases and research institutes as well as optimizing and reorganizing resources through mergers and sustainability acquisitions of some large companies, Company A has helped digital transformation. Its return on equity rose [19]. And in the following years, it has been stable at around 26%, not as volatile as the industry average. This indicates that the net assets injected by Group A after digital transformation can obtain more stable profits, and it also indicates that digital transformation can help the company further integrate assets to a certain extent.

Secondly, net profit margin on sales refers to the comparative relationship between net profit and sales revenue, which is used to measure the ability of enterprises to obtain sales revenue in a certain period.

As can be seen from Figure 4, compared with Group A before its digital transformation, the growth rate of gross margin was significantly accelerated in 2013 and was always in a state of steady growth. However, it fell in 2017, when the year-on-year growth rate of Company A's total operating revenue and costs was more than 50%, but the actual growth rate of operating expenses was about 5% higher than that of operating revenue. There are two reasons for this phenomenon: first, in 2017, China's home appliance industry is actively seeking online marketing channels, and the iterative demand for new products promotes the increase of revenue and cost of Company A's main business [20]. The second is also influenced by acquisitions. After the acquisition, the company's main business gross profit margin is less than 15%. These two reasons together lead to Company A's gross profit margin in 2017 lower than that in 2016. In the whole range, the increase or decrease of net return rate is basically the same as the gross margin. In 2017, the price of raw materials for home appliances rose sharply. In addition, the merger and acquisition at this stage increased expenses during the period, leading to a slight increase in net profit and a year-on-year decline in net interest rate.

Then the net profit margin on sales of Company A is compared with the industry average. As can be seen from Figure 5, net profit margin on sales was always lower than the industry average before 2014. In 2014, it exceeded the industry average and opened a gap with the industry average. From 2015 to 2016, it put forward the dual-intelligence strategy, which made the net profit margin on sales rise to 9.97%, 70% higher than the same period in 2010. In 2017, it was still affected by Company A's large-scale investment and acquisition, resulting in a sharp rise in costs and a sharp drop in net profit margin on sales [21]. However, in 2018, when the overall industry average level declined, Group A did not decline, but there was a big improvement, which indicates that after the digital transformation, Group A's profit stability gradually enhanced.

### 4.2. Operation Capacity Analysis

This article analyzes the operation capacity of Group A before and after digital transformation through inventory turnover and accounts receivable turnover.

First, inventory turnover is the ability of inventory to be converted into cash. As shown in Figure 6, a longitudinal comparison shows that the inventory turnover of Company A has been greatly improved after 2013, which is mainly due to the change of production and marketing mode of Group A during this period, which greatly reduces inventory pressure and optimizes inventory management through digital transformation. From 2013 to 2016, the inventory of Company A has been maintained at about 15 billion yuan. In 2015, due to the recession of domestic economy, the inventory was reduced by one third. Therefore, the inventory turnover speed of Company A will naturally improve under the condition of small inventory scale and steady increase of operating cost [22]. Since 2017, Company A's inventory scale has been better controlled, and in 2018, under the premise of rapid increase in sales volume and expansion of business scope, Group A's inventory control level is still quite high. However, due to the influence of the previous two years, the inventory backlog in 2016 was serious, resulting in a large difference between the average inventory balance in 2017 and 2018, resulting in a decline in the inventory turnover rate. In general, the liquidity of Company A's inventory has always been far ahead in the industry. Although there are some fluctuations in liquidity purely on the surface of the data, in fact, Company A has done a good job in inventory management. Through digital transformation, Group A can maintain the balance of inventory quantity in the continuous expansion of business development and reduce the company's operational risks to a certain extent [23].

A horizontal comparison between the inventory turnover rate of Group A and the industry average shows that, as shown in Figure 7, the inventory turnover rate of Company A was always slightly lower than the industry average before the transformation. However, since 2012, Company A began to adopt the mode of “sales” in inventory management. In the case of transparent all-channel inventory and cooperative management of entity enterprises, Company A constructed all-channel inventory sharing and realized the system's autonomous adjustment of inventory level by opening up the information flow of collaborative warehouses. Through the implementation of the order management mode, its inventory turnover rate increased to 8.87% in 2016, and it gradually exceeded the average level of the household appliance industry [24]. It can also be obviously found in Figure 7 that after digital transformation, the growth range of inventory turnover of Group A gradually increases, and the difference between Group A and the industry average also gradually expands. This shows that the inventory management of Group A is optimized through digital transformation, and the inventory turnover rate is improved, thus enhancing the operating strength of the company.

Secondly, accounts receivable turnover can be used to reflect the ability of enterprises to cash accounts receivable. Through the observation of the whole range, Company A's accounts receivable turnover has a great change. In 2012, the turnover of Group A had a slight decline and was even exceeded by the industry average, but it was improved immediately after the transformation. In particular, during 2016-2017, as Company A entered the digital 2.0 stage, it effectively reduced the credit sales business through online channels. In addition, the improvement of Company A's overall operating efficiency has shortened the delivery time of products and accelerated the collection speed of enterprises, so that the cash turnover of Company A's receivables can continue to improve and maintain a leading position in the whole industry. In general, through the evaluation of Group A's accounts receivable liquidity in the whole analysis region, it is found that it has been improving to a considerable extent, which not only alleviates the company's operating financing pressure, but also improves the company's short-term repayment ability.

Then compared with the same industry. As can be seen from Figure 8, before 2013, the receivables turnover rate of Company A was not very stable, with ups and downs, and showed a trend lower than the industry average [25]. After Group A has adopted comprehensive digital sales and improved the online trading platform, the turnover speed of its receivables has exceeded the industry average, which indicates that through the application of digital technology, Group A's ability to realize receivables has been improved and the enterprise has also been promoted to develop in a better direction.

### 4.3. Solvency Analysis

This article chooses asset-liability ratio and liquidity ratio to analyze the solvency of Group A.

The asset-liability ratio mainly refers to the ratio of total liabilities to total assets. The higher the ratio, the poorer the company's ability to repay arrears. Generally speaking, the asset-liability ratio should be between 40% and 60%.  Figure 9 shows that the asset-liability ratio of Group A showed a downward trend before 2017, but in the years 2017-2020, it always exceeded the average level of the industry, and almost reached 70%. In this case, it is very unfavorable for the company, because the company cannot repay the maturing debt, it needs to bear more interest costs, which damages the rights and interests of shareholders. Meanwhile, the company will face more risks, and the maturity of debt at different times will directly affect the company's capital flow. High debt ratio will make it difficult for the company to use debt financing to meet the needs of funds.

A horizontal comparison of Group A's asset-liability ratio with its competitors and the average value of the industry shows that the asset-liability ratio of Company A before 2016 is generally lower than the average value of the industry. In addition, the enterprise is still in the period of continuous development, and its asset-liability ratio can be maintained below 60% for a long time, which to some extent reflects the good capital chain operation of Company A. Since 2016, the average asset-liability ratio of competitors and the industry has been declining, indicating that its asset structure is optimizing. However, Company A keeps rising after the acquisition, and the corresponding financial risks also rise. Therefore, it can be seen that Company A's digital transformation has not kept its long-term solvency in good condition. All in all, there is still a lot of room for improvement in Company A's long-term solvency.

Second, the current ratio is used to show a company's ability to repay short-term debt. Generally speaking, the higher the ratio, the stronger the liquidity of the assets, and the stronger the short-term solvency.

As can be seen from Figure 10, the growth trend of liquidity ratio and quick ratio of Group A in the whole range is roughly the same. There was a slight decline in 2011-2012. Subsequently, in 2013, due to the continuous expansion of online channels, the credit sales business gradually decreased, and the working capital of enterprises increased, which almost showed a steady growth in the following years [26]. Meanwhile, by comparing the liquidity ratio between Group A and the industry average, it is found that Company A has not reached the industry average level before 2015. With the improvement of the time and intensity of digital transformation, the business performance improved [27]. After 2015, it began to exceed the industry average and gradually separated. In general, the short-term solvency of Company A has improved after digital transformation.

### 4.4. Growth Ability Analysis

This article selects the growth rate of net profit. The larger the index value is, the better the future development prospect of the enterprise is.

As far as shareholders are concerned, net profit can better reflect their own investment reporting.  Figure 11 shows that during the whole period, its net profit grew faster than its operating income. Especially after the digital transformation, the growth rate of net profit increased significantly. Despite the economic downturn, fierce competition in the home appliance industry and corporate acquisitions, the year-on-year growth rate of net profit was maintained at about 17%. From this point of view, Group A's adaptability to the outside world has been continuously enhanced in the transformation process, and the company's internal management system has also been improved to some extent, which helps the sustainable development of the enterprise.

Meanwhile, the net profit growth rate of Company A is compared with the average level of the industry. As can be seen from Figure 12, the growth rate of Company A's net profit dropped sharply from 88% to negative value before 2013. After digital transformation, IT systems are restructured, administrative costs are reduced, and operating revenues are increased. The net profit growth rate of Group A has risen in a fluctuating manner and has exceeded the average of the household appliance industry, which means that the digital transformation of Company A is playing a positive role in the profitability of the enterprise, but it is not stable enough. After 2015, the growth rate of Company A's net profit has been hovering between 16% and 17%, mainly because it has reached a saturation level in the traditional business sector and the profit space is not large, which is also an important reason for Company A to take the initiative to carry out digital transformation. In 2017, Group A increased investment in research and development, improved research and development capabilities, and increased investment in robotics, intelligence, and other sectors. However, the current profitability is not known, and it takes time to integrate and verify. In general, the digital transformation of Company A is beneficial to the growth and development of the enterprise, but the effect is not obvious, and more time is needed to test.

It is difficult to obtain a comprehensive evaluation by analyzing the effect of digital transformation separately from various indicators of financial dimension. Therefore, through comprehensive analysis of financial performance, this article combines all indicator systems together to comprehensively evaluate the digital transformation of Group A.

First, establish the company's comprehensive financial performance analysis system and measure it. In the four ability data of company debt paying, operation, profitability and growth, two typical indicators are selected to conduct comprehensive evaluation and analysis on the digital transformation case of Company A. Then, according to the Operation Rules for Company Performance Evaluation (Revised Edition), weight is given to the selected index system to establish Company A's exclusive comprehensive evaluation framework. The indicators after the transformation are evaluated comprehensively to determine the final score. The specific basis for selecting the index system is as follows: in terms of solvency, the asset-liability ratio and current ratio are selected to measure. In terms of operating capacity, accounts receivable turnover and inventory turnover rate indices are selected to measure. In terms of profit level, the article selects the return on equity which can reflect the effective use effect of the owner's investment funds and the sales net profit which can best reflect the effect of sales revenue. In terms of growth ability, operating income growth rate and net profit growth rate are adopted. Based on the above analysis, the selected indicators and weights are sorted into a table, as shown in Table 1.

The comprehensive financial performance evaluation in this article selects 2012 to 2020 as the evaluation period, and the index values are shown in Table 2 below:

This article uses the average evaluation index data of the household appliance industry as the reference value, as detailed in Table 3.

Divide Table 2 and Table 3 to obtain the standard coefficient relative to each financial index of Group A from 2012 to 2020. See Table 4 for the specific data.

The standard coefficient value of the above table is multiplied by the given scoring weight to calculate the data of eight evaluation items, and the data results are all added up. See Table 5 for the specific data.

Then, the comprehensive score of financial performance is analyzed. As can be seen from Figure 13, the comprehensive score of Group A's financial performance in 2012 was very low, and neither the growth ability nor the business strength achieved the desired effect. Under such circumstances, Company A began to implement digital transformation, the overall IT system was comprehensively reconstructed, and the new mode of “sales to production” was implemented in the inventory management mode. By 2013, the financial performance composite score had increased significantly. Although in 2015, due to the decline of net profit growth rate, the comprehensive score of financial performance fell. However, Group A immediately increased the intensity of digital transformation to recover the situation of falling profits. Since 2016, the continuous improvement of profitability and growth ability of Group A has promoted the overall positive trend of financial performance. The comprehensive score of financial performance is always above the standard score. Through the comprehensive analysis of financial performance, it is concluded that the digital transformation of Group A has been effective and the enterprise value has increased significantly.

## 5. Conclusion

In order to cope with the impact of digital technology, adapt to changes in the external environment, and ensure its own stable development, Group A, as a traditional household appliance manufacturing enterprise, uses various digital technologies to transform and upgrade its links and realize the digitalization of the enterprise as a whole. This article explores the path and mechanism of Group A's digital transformation and analyzes the performance of Group A before and after the transformation by using relevant indicators. There are four main reasons for Group A's digital transformation: to meet the needs of the development of the digital economy era, to support national policies, to enhance the core competitiveness of the enterprise, to reduce product costs, and to meet the diversified needs of customers. Digital transformation can improve enterprise performance. In this article, the performance of Group A before and after digital transformation is comparatively analyzed from the four dimensions of the balanced scorecard. The results show that since the digital transformation began in 2012, Group A has improved its profitability, operation and growth capacity, and maintained a leading position in the entire household appliance industry.

## Figures and Tables

**Figure 1:** Motivation of enterprise digital transformation.

**Figure 2:** T+3 mode of Group A.

**Figure 3:** Comparison of ROE and industry average of Group A from 2010 to 2020.

**Figure 4:** Changes of Group A's gross profit margin and net profit margin on sales from 2010 to 2020.

**Figure 5:** Comparison of Group A's net profit margin on sales and industry average from 2010 to 2020.

**Figure 6:** Inventory turnover of Group A from 2010 to 2020.

**Figure 7:** Comparison of Group A's inventory turnover rate and industry average from 2010 to 2020.

**Figure 8:** Accounts receivable turnover rate and industry average of Group A from 2010 to 2020.

**Figure 9:** Comparison of the average asset-liability ratio of Group A, its competitors, and the industry from 2010 to 2020.

**Figure 10:** Current ratio and quick ratio of Group A from 2010 to 2020.

**Figure 11:** Year-on-year growth of Net profit and operating revenue of MideGroup A from 2010 to 2020.

**Figure 12:** Group A's net profit growth rate and industry average from 2010 to 2020.

**Figure 13:** Change trend of A Group's comprehensive score of financial performance from 2012 to 2020.

**Table 1:** Comprehensive analysis index table of MideGroup A financial performance.

Evaluation index	Selected indicators	Weight (%)
Debt paying ability	Asset-liability ratio	12
	Current ratio	8

Operation ability	Accounts receivable turnover	9
	Inventory turnover	9

Profitability	Return on equity	25
	Net profit margin on sales	13

Growth ability	Growth rate of operating income	12
	Net profit growth rate	12

**Table 2:** Index values of Group A from 2012 to 2020.

Year	2012	2013	2014	2015	2016	2017	2018	2019	2020
Asset-liability ratio (%)	37.8	40.31	38.02	43.49	40.43	33.42	35.06	35.6	34.47
Current ratio	1.09	1.15	1.18	1.3	1.35	1.43	1.4	1.5	1.31
Accounts receivable turnover (times)	4.84	5.47	5.84	5.57	7.21	9.77	8.61	10.05	10.99
Inventory turnover (times)	5.35	6.5	6.99	8.06	8.87	8.01	6.37	6.38	6.7
Return on equity (%)	23.92	24.87	29.49	29.06	26.88	25.88	25.66	26.43	24.95
Net profit margin on sales (%)	5.99	6.86	8.22	9.84	9.97	7.73	8.34	9.09	9.68
Growth rate of operating revenue (%)	-23.41	18.06	17.36	-2.08	14.71	51.35	8.23	6.71	2.27
Net profit growth rate (%)	-5.5	63.15	97.5	20.99	15.56	17.7	17.05	19.68	12.44

**Table 3:** Average index value table of home appliance manufacturing industry from 2012 to 2020.

Year	2012	2013	2014	2015	2016	2017	2018	2019	2020
Asset-liability ratio (%)	35.74	36.51	38.14	40.95	38.18	37.34	38.67	39.07	39.92
Current ratio	1.28	1.28	1.29	1.27	1.25	1.3	1.32	1.32	1.32
Accounts receivable turnover (times)	6.86	4.37	4.1	2.99	3.1	4.89	5.06	5.21	4.34
Inventory turnover (times)	5.18	5.72	6.47	6.66	6.56	6.34	6.03	5.8	5.78
Return on equity (%)	15.91	18.66	19.91	16.1	18.29	20.15	15.2	15.98	14.7
Net profit margin on sales (%)	6.25	7.06	7.84	8.59	8.87	7.22	7.11	7.95	8.02
Growth rate of operating revenue (%)	1.53	15.47	15.3	-12.54	18.96	41.59	18.07	5.33	-2.75
Net profit growth rate (%)	18.99	46.04	51.87	-3.28	18.7	33.19	14.12	7.86	3.47

**Table 4:** Index standard coefficients of Group A from 2012 to 2020.

Year	2012	2013	2014	2015	2016	2017	2018	2019	2020
Asset-liability ratio (%)	1.06	1.1	1	1.06	1.06	0.9	0.91	0.91	0.86
Current ratio	0.85	0.9	0.91	1.02	1.08	1.1	1.06	1.14	0.99
Accounts receivable turnover (times)	0.71	1.25	1.42	1.86	2.33	2	1.7	1.93	2.53
Inventory turnover (times)	1.03	1.14	1.08	1.21	1.35	1.26	1.06	1.1	1.16
Return on equity (%)	1.5	1.33	1.48	1.8	1.47	1.28	1.69	1.65	1.7
Net profit margin on sales (%)	0.96	0.97	1.05	1.15	1.12	1.07	1.17	1.14	1.21
Growth rate of operating revenue (%)	-15.3	1.17	1.13	0.17	0.78	1.23	0.46	1.26	-0.83
Net profit growth rate (%)	-0.29	1.37	1.88	-6.4	0.83	0.53	1.21	2.5	3.59

**Table 5:** Score table of Group A's four competencies and comprehensive performance from 2012 to 2020.

Year	2012	2013	2014	2015	2016	2017	2018	2019	2020
Solvency score	19.52	20.4	19.28	20.88	21.36	19.6	19.4	20.04	18.24
Operational capability score	15.66	21.51	22.5	27.63	33.12	29.34	24.84	27.27	33.21
Profitability score	49.98	45.86	50.65	59.95	51.31	45.91	57.46	56.07	58.23
Growth ability score	-187.08	30.48	36.12	-74.76	19.32	21.12	20.04	45.12	33.12
Solvency score	19.52	20.4	19.28	20.88	21.36	19.6	19.4	20.04	18.24
Comprehensive score of financial performance	-101.92	118.25	128.55	33.7	125.11	115.97	121.74	148.5	142.8

## Data Availability

The data that support the findings of this study are available from the corresponding author upon reasonable request.
